The article "Lack of specificity of antibodies raised against CLN3, the lysosomal/endosomal transmembrane protein mutated in juvenile Batten disease" was published in 2017. Journal: Biosci Rep.

# Lack of specificity of antibodies raised against CLN3, the lysosomal/endosomal transmembrane protein mutated in juvenile Batten disease

**DOI:** 10.1042/BSR20171229

**Published:** 2017-11-23

**Authors:** Tarah Nelson, David A. Pearce, Attila D. Kovács

**Affiliations:** 1 Pediatric and Rare Diseases Group, Sanford Research, Sioux Falls, South Dakota 57104, U.S.A.; 2 Department of Pediatrics, Sanford School of Medicine, University of South Dakota Sioux Falls, South Dakota 57104, U.S.A.

**Keywords:** anti-CLN3 antibodies, Batten disease, Neuronal Ceroid Lipofuscinosestein, transmembrane protein

## Abstract

Juvenile CLN3 (Batten) disease, a fatal, childhood neurodegenerative disorder, results from mutations in the *CLN3* gene encoding a lysosomal/endosomal transmembrane protein. The exact physiological function of CLN3 is still unknown and it is unclear how *CLN3* mutations lead to selective neurodegeneration. To study the tissue expression and subcellular localization of the CLN3 protein, a number of anti-CLN3 antibodies have been generated using either the whole CLN3 protein or short peptides from CLN3 for immunization. The specificity of these antibodies, however, has never been tested properly. Using immunoblot experiments, we show that commercially available or researcher-generated anti-CLN3 antibodies lack specificity: they detect the same protein bands in wild-type (WT) and *Cln3^−/−^* mouse brain and kidney extracts prepared with different detergents, in membrane proteins isolated from the cerebellum, cerebral hemisphere and kidney of WT and *Cln3^−/−^* mice, in cell extracts of WT and *Cln3^−/−^* mouse embryonic fibroblast cultures, and in lysates of BHK cells lacking or overexpressing human CLN3. Protein BLAST searches with sequences from peptides used to generate anti-CLN3 antibodies identified short motifs present in a number of different mouse and human proteins, providing a plausible explanation for the lack of specificity of anti-CLN3 antibodies. Our data provide evidence that immunization against a transmembrane protein with low to medium expression level does not necessarily generate specific antibodies. Because of the possible cross-reactivity to other proteins, the specificity of an antibody should always be checked using tissue samples from an appropriate knock-out animal or using knock-out cells.

## Introduction

Neuronal ceroid lipofuscinoses, also known as Batten disease, are a group of inherited lysosomal storage disorders with progressive neurodegeneration mostly affecting children. The most common form, juvenile CLN3 (Batten) disease is caused by mutations in the *CLN3* gene [1,2]. The disease begins between 4 and 10 years of age and the common symptoms are visual impairment with retinal degeneration that eventually leads to complete blindness, seizures, and progressive motor and cognitive decline due to widespread neurodegeneration [3]. Most patients die in their 20s.

The article "Lack of specificity of antibodies raised against CLN3, the lysosomal/endosomal transmembrane protein mutated in juvenile Batten disease" was published in 2017. Journal: Biosci Rep.

The *CLN3* gene encodes a 438 amino-acid integral membrane protein with six transmembrane domains, the N- and C-termini are both found in the cytosol [1,4]. CLN3 contains three lysosomal localization motifs: two dileucine sorting motifs in the cytosolic internal loop and an acidic patch found in the C-terminus [5–7]. CLN3 has two glycosylation sites at asparagines 71 and 85 [8], its C-terminus is farnesylated [8–10], and CLN3 may also be phosphorylated at serine and threonine residues [11–13]. The exact physiological function of the CLN3 protein is still unknown. Studies in yeast, mammalian and human cells, and in mice suggest the involvement of CLN3 in various cellular processes including regulation of lysosomal pH [14–17] and arginine transport [18,19], endocytosis and endosomal trafficking [20–22], autophagy [17,23], protein transport between the *trans*-Golgi and endosomes [24–26], proliferation [27–31], and apoptosis [29–32]. It is unclear, however, in which process CLN3 has a real functional role and which process is affected as a secondary consequence of its primary function.

To study the tissue expression and subcellular localization of the CLN3 protein, several anti-CLN3 antibodies have been generated using either the whole CLN3 protein or short peptides from CLN3 for immunization [7,8,33–40]. The specificity of these antibodies, however, has never been tested properly. In the present study, we tested commercially available and researcher-generated anti-CLN3 antibodies in immunoblot experiments using protein extracts from wild-type (WT) and *Cln3^−/−^* mouse tissues. Our results show that the anti-CLN3 antibodies lack specificity, they detect the same protein bands in WT and *Cln3^−/−^* samples, indicating that immunization against a transmembrane protein with low to medium expression level does not necessarily generate specific antibodies.

## Materials and methods

### Animals

In the present study, 129S6/SvEv WT male mice and homozygous *Cln3*-knockout (*Cln3^−/−^*) male mice [41] inbred on the129S6/SvEv background were used. All procedures were carried out according to the guidelines of the Animal Welfare Act, NIH policies, and were approved by the Sanford Research Animal Care and Use Committee.

### Antibodies

The anti-CLN3 antibodies used in the present study are described in Table 1. The rabbit anti-myc-tag antibody (2272) was obtained from Cell Signaling Technologies (Danvers, MA). The horseradish peroxidase-conjugated donkey anti-rabbit IgG F(ab’)_2_ fragment (NA9340) and sheep anti-mouse IgG (NA931) (Amersham ECL antibodies) were purchased from GE Healthcare Life Sciences (Piscataway, NJ). The mouse anti-goat IgG coupled to horseradish peroxidase (sc-2354) was from Santa Cruz Biotechnology (Santa Cruz, CA).

The article "Lack of specificity of antibodies raised against CLN3, the lysosomal/endosomal transmembrane protein mutated in juvenile Batten disease" was published in 2017. Journal: Biosci Rep.

**Table 1:** Anti-CLN3 antibodies used in the present study

Source	Description	Immunogen	Purity	Species reactivity	Recommended dilution for immunoblotting	Dilution used in the study
Abnova	Rabbit polyclonal D01P	Full-length human CLN3	Immunogen affinity purified	Human, mouse	1:500–1:1000	1:500
Abnova	Mouse monoclonal M03	Full-length recombinant human CLN3 with GST tag	Purified IgG	Human, other species not tested	1:200–1:1000	1:500
Abcam	Rabbit polyclonal ab75959	A synthetic peptide derived from within residues 400–438 of human CLN3	Immunogen affinity purified	Human, mouse, rat	1:700	1:700
Abcam	Rabbit polyclonal ab87438	A synthetic peptide derived from within residues 50–150 of human CLN3	Immunogen affinity purified	Mouse	1:1000	1:1000
Santa Cruz	Goat polyclonal D-20	A synthetic peptide mapping at the N-terminus of mouse CLN3	Immunogen affinity purified	Mouse, rat, human	1:100–1:1000	1:100
Santa Cruz	Goat polyclonal P-20	A synthetic peptide mapping within an internal region of mouse CLN3	Immunogen affinity purified	Mouse, rat	1:100–1:1000	1:100
Santa Cruz	Goat polyclonal C-16	A synthetic peptide mapping near the C-terminus of human CLN3	Immunogen affinity purified	Mouse, rat, human	1:100–1:1000	1:100
Anu Jalanko’s group, Finland	Rabbit polyclonal m385	A synthetic peptide corresponding to amino acids 242–258 of mouse CLN3	Immunogen affinity purified	Mouse, human	1:500–1:1000	1:1000
Our group	Rabbit polyclonal 9033	A synthetic peptide corresponding to amino acids 5–19 of mouse CLN3	Serum	Mouse	1:50–1:500	1:100

### Protein extract preparation

#### Surface cross-linked cerebellum and cortex tissue samples from 1-month-old WT and Cln3^−/−^ male mice

Protein extracts were prepared as we previously described [42,43]. Briefly, the surface cross-linked tissue slices in 1.5-ml microtubes were homogenized by sonication in ice-cold lysis buffer [25 mM HEPES (pH 7.4), 500 mM NaCl, 2 mM EDTA, 20 mM NaF, 1 mM sodium orthovanadate, 0.1% NP-40 substitute, 1 mM DTT, protease inhibitor cocktail, and phosphatase inhibitor cocktail (Sigma)]. The microtubes were vortexed for 8 s and then centrifuged at 20000 ***g*** for 2 min at 4°C. The supernatants were transferred into new precooled microtubes and total protein concentration of the lysates was determined by the Pierce 660-nm protein assay (Pierce, Rockford, IL). The samples were aliquoted and stored at −80°C until further analysis.

The article "Lack of specificity of antibodies raised against CLN3, the lysosomal/endosomal transmembrane protein mutated in juvenile Batten disease" was published in 2017. Journal: Biosci Rep.

#### Cerebral hemisphere and kidney from 254-day-old WT and 285-day-old Cln3^−/−^ male mice

Protein extracts from the right cerebral hemisphere and the kidney were prepared in a lysis buffer containing 50 mM sodium phosphate (pH 7.4), 1% *n*-dodecyl-β-D-maltopyranoside (DDM), 1 mM DTT, protease inhibitor cocktail, and phosphatase inhibitor cocktail (Sigma). The cerebral hemisphere and kidney were cut into small pieces with a razor blade and homogenized on ice with the lysis buffer (300 µl/tube) in 1.5-ml microtubes using pellet pestles. The tubes were then incubated at room temperature for 3 min, vortexed for 12 s, and incubated at room temperature for an additional 2 min. Then, the lysates were flesh frozen and thawed three times to shear genomic DNA. Finally, the samples were centrifuged at 20000 ***g*** for 5 min at 4°C. The supernatants were transferred into new precooled microtubes and total protein concentration of the lysates was determined by the Pierce 660-nm protein assay (Pierce, Rockford, IL). The samples were aliquoted and stored at −80°C until further analysis.

#### Baby hamster kidney (BHK) cells and mouse embryonic fibroblast cultures

Protein samples were prepared from equal numbers of cells grown in 10-cm culture dishes (Corning Inc., Corning, NY). Cells were washed three times with ice-cold PBS, scraped into ice-cold PBS (1 ml/culture dish), transferred into 2-ml tubes, and centrifuged at 200 ***g*** for 5 min at 4°C. The cell pellets were suspended in ice-cold lysis buffer containing either DDM [50 mM sodium phosphate (pH 7.4), 1% DDM, 1 mM DTT, protease inhibitor cocktail, and phosphatase inhibitor cocktail (Sigma)] or Triton X-100 [50 mM Tris/HCl (pH 7.5), 300 mM NaCl, 5 mM EDTA, 1% Triton X-100, 1 mM DTT, protease inhibitor cocktail, and phosphatase inhibitor cocktail (Sigma)], vortexed vigorously for 10 s, and incubated on ice for 30 min. The tubes were then centrifuged at 20000 ***g*** for 10 min at 4°C. The supernatants were transferred into new precooled 1.5-ml microtubes and total protein concentration of the lysates was determined by the Pierce 660-nm protein assay (Pierce, Rockford, IL). The samples were aliquoted and stored at −80°C until further analysis.

### Membrane protein isolation

Membrane proteins were isolated from the kidney, cerebellum, and the left cerebral hemisphere of 254-day-old WT and 285-day-old *Cln3^−/−^* male mice, and from WT and *Cln3^−/−^* embryonic fibroblast cultures using the BioVision Membrane Protein Extraction Kit (BioVision, Milpitas, CA; catalog # K268-50) according to the manufacturer’s protocol. Isolated membrane proteins were dissolved in PBS containing 0.5% Triton X-100, 1 mM DTT, protease inhibitor cocktail, and phosphatase inhibitor cocktail (Sigma). Concentration of the isolated membrane proteins was determined by the Pierce 660-nm protein assay (Pierce, Rockford, IL). The samples were aliquoted and stored at −80°C until further analysis.

The article "Lack of specificity of antibodies raised against CLN3, the lysosomal/endosomal transmembrane protein mutated in juvenile Batten disease" was published in 2017. Journal: Biosci Rep.

### Cell culture and transfection

WT and *Cln3^−/−^* mouse embryonic fibroblast cultures were prepared and maintained as we previously described [44]. BHK cells were cultured as we described previously [45]. BHK cells were transfected with either a pBudCE4.1 plasmid expressing N-terminally myc-tagged human CLN3 or the empty pBudCE4.1 plasmid (Thermo Fisher Scientific, Waltham, MA) using Lipofectamine 2000 (Thermo Fisher Scientific, Waltham, MA) according to the manufacturer’s protocol. Thirty-six hours after transfection, BHK cells were lysed in a lysis buffer containing 1% DDM as described above.

### Immunoblotting

Samples (60-µg total protein) were incubated in reducing sample buffer (without urea, Figure 1, or with 4 M urea, Figures 1–5) for 10 min at 100°C or for 15 min at 65°C (Figure 1) or for 30 min at 37°C (Figures 1–5), then loaded and electrophoresed on 10% Tris/HCl SDS gels under reducing conditions. After the electrophoretic separation, proteins were transferred onto nitrocellulose or PVDF membranes (Millipore, Billerica, MA) using the standard wet transfer method at 100 V for 80 min. Membranes were rinsed twice with ultrapure water and blocked with 5% nonfat dry milk in Tris-buffered salt solution containing 0.1% Tween-20 (TBS-T) for 2 h at room temperature. Membranes were then incubated with the anti-CLN3 antibodies (recommended and used dilutions are listed in Table 1) or the anti-myc antibody (1:1000) in TBS-T containing 5% nonfat dry milk overnight at 4°C. Membranes were rinsed twice with ultrapure water, washed with TBS-T (first for 10 min, then three times for 5 min each), and incubated with the appropriate horseradish peroxidase-conjugated secondary antibody [donkey anti-rabbit IgG F(ab’)_2_ fragment (1:10000), sheep anti-mouse IgG (1:5000), or mouse anti-goat IgG (1:5000)] for 1.5 h at room temperature. Membranes were then rinsed twice with ultrapure water and washed with TBS-T (first for 10 min then four times for 5 min each). After being rinsed twice with ultrapure water, membranes were incubated in Amersham ECL Plus chemiluminescence detection reagent (GE Healthcare Life Sciences, Piscataway, NJ) for 5 min and imaged using a Biospectrum 500 Imaging System (UVP, Upland, CA).

**Figure 1:** Anti-CLN3 antibodies detect the same protein bands in wild-type (WT) and *Cln3^−/−^* mouse brain extracts Three different anti-CLN3 antibodies [Abnova rabbit anti-CLN3 (D01P), Abnova mouse anti-CLN3 (M03), and Abcam rabbit anti-CLN3 (ab75959)] were tested in immunoblot experiments using protein extracts of surface cross-linked cerebellum and cortex tissue samples from 1-month-old WT and *Cln3^−/−^* male mice. Protein extracts were prepared by sonication in a lysis buffer containing 500 mM NaCl, 0.1% NP-40 substitute and protease, and phosphatase inhibitor cocktails. Sixty micrograms of protein were loaded in each lane of SDS-containing 10% polyacrylamide gels. Prior to loading, samples were treated as indicated in reducing sample buffer without or with 4 M urea. After the electrophoretic separation, proteins were transferred onto nitrocellulose membranes and probed with the anti-CLN3 antibodies (Abnova rabbit, 1:500; Abnova mouse, 1:500; Abcam rabbit, 1:700); M.W. marker: PageRuler Plus (Thermo Fisher Scientific). The immunoblots shown are representative of two separate experiments.

The article "Lack of specificity of antibodies raised against CLN3, the lysosomal/endosomal transmembrane protein mutated in juvenile Batten disease" was published in 2017. Journal: Biosci Rep.

In the case of mouse embryonic fibroblast culture extracts (Figure 4), the membranes were blocked with 1% nonfat dry milk in TBS-T and incubated with the primary and secondary antibodies in 1% nonfat dry milk in TBS-T.

## Results

The *Cln3* gene is widely expressed in the brain and kidney [36,46] and has important physiological functions in these tissues [33,41,46]. To examine if commercially available and researcher-generated anti-CLN3 antibodies recognize the endogenous CLN3 protein, we utilized brain and kidney extracts from WT and *Cln3^−/−^* mice in immunoblot experiments. Endogenous CLN3 should appear as a distinct ∼48-kDa band only present in WT samples. Table 1 lists the anti-CLN3 antibodies used in experiments presented in Figures 1–5.

First, we tested a rabbit polyclonal antibody raised against the full-length human CLN3 (Abnova, recommended dilution: 1:500–1:1000; dilution used in the present study: 1:500), a mouse monoclonal antibody raised against the full-length human CLN3 with a glutathione S-transferase (GST) tag (Abnova, recommended dilution: 1:200–1:1000; dilution used in the present study: 1:500), and a rabbit polyclonal antibody produced against a synthetic peptide derived from within residues 400–438 of human CLN3 (Abcam; applied in the recommended dilution of 1:700) using protein extracts of surface cross-linked cerebellum and cortex tissue samples from 1-month-old WT and *Cln3^−/−^* male mice. These protein extracts were prepared by sonication in a lysis buffer containing 500 mM NaCl and 0.1% NP-40 substitute, and we have used aliquots of these samples in immunoblot experiments to successfully measure the intracellular and surface expression of AMPA and NMDA receptor subunits [43]. To optimize the solubilization of hydrophobic membrane proteins (such as CLN3) for gel electrophoresis, protein extracts (60 µg) were incubated with SDS/PAGE reducing sample buffer at various temperatures (37°C for 30 min, 65°C for 15 min, and 100°C for 10 min), and urea-containing sample buffer (4 M, 65°C for 15 min) was also tested. Urea is a chaotropic agent and prevents aggregation of hydrophobic membrane proteins. As Figure 1 shows, none of the three anti-CLN3 antibodies detected a specific band in WT brain extracts under any of the sample processing conditions applied.

The article "Lack of specificity of antibodies raised against CLN3, the lysosomal/endosomal transmembrane protein mutated in juvenile Batten disease" was published in 2017. Journal: Biosci Rep.

DDM has been found to be a superior detergent for solubilizing hydrophobic membrane proteins [47–49]. We have previously found that in baby hamster kidney (BHK) cells stably expressing myc-tagged human CLN3, lysis buffer containing 1% DDM extracted myc-CLN3 more efficiently than lysis buffer containing 1% Triton X-100 [45]. Therefore, we prepared protein extracts with 1% DDM-containing lysis buffer from the brain (right cerebral hemisphere) and kidney of adult WT and *Cln3^−/−^* mice, and tested the Abnova rabbit and mouse (1:500), and Abcam rabbit (1:700) anti-CLN3 antibodies on these samples. In the same experiments, we also used extracts of BHK cells transfected either with a pBudCE4.1 plasmid expressing myc-tagged human CLN3 or with the empty plasmid; BHK cell extracts were also prepared with 1% DDM-containing lysis buffer. Prior to loading on SDS-containing 10% polyacrylamide gels, the brain, kidney, and BHK cell extract samples (60 µg) were incubated at 37°C for 30 min in reducing sample buffer containing 4 M urea. The CMV (Cytomegalovirus) promoter in the pBudCE4.1 plasmid provided high-level expression of myc-CLN3 in BHK cells as detected by an anti-myc tag antibody (Figure 2, bottom right blot). The three anti-CLN3 antibodies, however, did not detect myc-CLN3 in BHK cell extracts, or any specific band in the WT brain and kidney extracts compared with *Cln3^−/−^* samples (Figure 2, top two and bottom left blots).

**Figure 2:** Anti-CLN3 antibodies do not detect CLN3 in mouse tissue extracts prepared with a special detergent or in BHK cells overexpressing human CLN3 Three different anti-CLN3 antibodies [Abnova rabbit anti-CLN3 (D01P), Abnova mouse anti-CLN3 (M03), and Abcam rabbit anti-CLN3 (ab75959)] were tested in immunoblot experiments using protein extracts prepared with the nonionic detergent, *n*-dodecyl-β-D-maltopyranoside (DDM), from the kidney and the right cerebral hemisphere (RCH) of 254-day-old WT and 285-day-old *Cln3^−/−^* male mice. Extracts of BHK cells transfected with either a plasmid overexpressing myc-tagged human CLN3 or the plasmid vector only were also used in these experiments. BHK cell extracts were prepared with 1% DDM-containing lysis buffer. Sixty micrograms of protein were loaded in each lane of SDS-containing 10% polyacrylamide gels. Prior to loading, samples were incubated at 37°C for 30 min in reducing sample buffer containing 4 M urea. After the electrophoretic separation, proteins were transferred onto nitrocellulose membranes and probed with the anti-CLN3 antibodies (Abnova rabbit, 1:500; Abnova mouse, 1:500; Abcam rabbit, 1:700). The mouse anti-myc antibody from Cell Signaling was used in a dilution of 1:1000; M.W. marker: PageRuler Plus (Thermo Fisher Scientific). The immunoblots shown are representative of two separate experiments.

The article "Lack of specificity of antibodies raised against CLN3, the lysosomal/endosomal transmembrane protein mutated in juvenile Batten disease" was published in 2017. Journal: Biosci Rep.

Although a relatively high amount of tissue extract (60-µg protein per lane) was loaded on the SDS-polyacrylamide gels, it was possible that the anti-CLN3 antibodies did not detect endogenous CLN3 because its tissue expression level is too low. To enrich for CLN3, we isolated membrane proteins from the brain (cerebellum and left cerebral hemisphere) and kidney of adult WT and *Cln3^−/−^* mice, and tested the Abnova rabbit and mouse (1:500), and Abcam rabbit (1:700) anti-CLN3 antibodies as well as three different Santa Cruz goat anti-CLN3 antibodies (recommended dilution: 1:100–1:1000; dilution used in the present study: 1:100) on these samples. Figure 3 shows that all six antibodies detected the same protein bands in WT samples as in *Cln3^−/−^* samples. The detected bands, however, varied among the antibodies and tissue types.

**Figure 3:** Anti-CLN3 antibodies do not detect a specific band in membrane protein samples isolated from the kidney, cerebellum, and cerebral hemisphere of WT mice Six different anti-CLN3 antibodies [Abnova rabbit anti-CLN3 (D01P), Abnova mouse anti-CLN3 (M03), Abcam rabbit anti-CLN3 (ab75959), Santa Cruz goat anti-CLN3 antibodies: C-16, P-20, and D-20] were tested in immunoblot experiments using membrane protein (M.P.) samples. Membrane proteins were isolated from the kidney, cerebellum, and the left cerebral hemisphere (LCH) of 254-day-old WT and 285-day-old *Cln3^−/−^* male mice using the BioVision Membrane Protein Extraction Kit. Sixty micrograms of protein were loaded in each lane of SDS-containing 10% polyacrylamide gels. Prior to loading, samples were incubated at 37°C for 30 min in reducing sample buffer containing 4 M urea. After the electrophoretic separation, proteins were transferred onto nitrocellulose membranes and probed with the anti-CLN3 antibodies (Abnova rabbit, 1:500; Abnova mouse, 1:500; Abcam rabbit, 1:700; all three Santa Cruz antibodies, 1:100); M.W. marker: PageRuler Plus (Thermo Fisher Scientific). The immunoblots shown are representative of two separate experiments.

The article "Lack of specificity of antibodies raised against CLN3, the lysosomal/endosomal transmembrane protein mutated in juvenile Batten disease" was published in 2017. Journal: Biosci Rep.

We also tested the Abnova rabbit and mouse (1:500), and Abcam rabbit (1:700) anti-CLN3 antibodies on cell lysates and isolated membrane proteins from WT and *Cln3^−/−^* mouse embryonic fibroblast cultures. Again, these three antibodies recognized the same bands in WT samples as in *Cln3^−/−^* samples (Figure 4).

**Figure 4:** Anti-CLN3 antibodies detect the same bands in protein extracts of WT and *Cln3^−/−^* mouse embryonic fibroblast cultures Three different anti-CLN3 antibodies [Abnova rabbit anti-CLN3 (D01P), Abnova mouse anti-CLN3 (M03), and Abcam rabbit anti-CLN3 (ab75959)] were tested in immunoblot experiments using cell lysates and isolated membrane proteins from WT and *Cln3^−/−^* mouse embryonic fibroblast cultures. Cell lysates were prepared with a lysis buffer containing either 1% Triton X-100 or 1% DDM. Membrane proteins were isolated using the BioVision Membrane Protein Extraction Kit. Sixty micrograms of protein were loaded in each lane of SDS-containing 10% polyacrylamide gels. Prior to loading, samples were incubated at 37°C for 30 min in reducing sample buffer containing 4 M urea. After the electrophoretic separation, proteins were transferred onto nitrocellulose membranes and probed with the anti-CLN3 antibodies (Abnova rabbit, 1:500; Abnova mouse, 1:500; Abcam rabbit, 1:700); M.W. marker: PageRuler Plus (Thermo Fisher Scientific). The immunoblots shown are representative of two separate experiments.

Figure 5 shows the immunoblot results with three additional anti-CLN3 antibodies. The 9033 rabbit anti-CLN3 serum was generated in our lab by immunizing with a peptide corresponding to amino acids 5–19 of mouse CLN3. This peptide was previously used by Ezaki et al. [50] to generate a rabbit anti-CLN3 antibody. The m385 rabbit anti-CLN3 antibody raised against a peptide with the amino acid sequence 242–258 of mouse CLN3 [36] was provided us by Dr Anu Jalanko (National Institute for Health and Welfare, Genomics and Biomarkers Unit, Helsinki, Finland; recommended dilution: 1:500–1:1000; dilution used in the present study: 1:1000). The Abcam rabbit anti-CLN3 antibody (ab87438; used in the recommended dilution of 1:1000) was raised against a synthetic peptide derived from within residues 50–150 of human CLN3. These antibodies were tested using isolated membrane proteins and protein extracts (1% DDM-containing lysis buffer) from the brain and kidney of WT and *Cln3^−/−^* mice. None of the three antibodies detected a specific band in WT samples that was missing in *Cln3^−/−^* samples (Figure 5).

**Figure 5:** Lack of specificity of three additional anti-CLN3 antibodies Three additional anti-CLN3 antibodies [9033 rabbit anti-CLN3 serum, m385 rabbit anti-CLN3, and Abcam rabbit anti-CLN3 (ab87438) antibodies] were tested in immunoblot experiments using tissue extracts and membrane protein (M.P.) samples. Membrane proteins were isolated from the kidney, cerebellum, and the left cerebral hemisphere (LCH) of 254-day-old WT and 285-day-old *Cln3^−/−^* male mice using the BioVision Membrane Protein Extraction Kit. Tissue extracts from the kidney and the right cerebral hemisphere (RCH) were prepared with a lysis buffer containing 1% DDM. Sixty micrograms of protein were loaded in each lane of SDS-containing 10% polyacrylamide gels. Prior to loading, samples were incubated at 37°C for 30 min in reducing sample buffer containing 4 M urea. After the electrophoretic separation, proteins were transferred onto a nitrocellulose membrane (9033) or PVDF membranes [m385 and Abcam (ab87438)], and the membranes were probed with the anti-CLN3 antibodies [9033, 1:400; m385, 1:1000; Abcam rabbit (ab87438), 1:1000]; M.W. markers: 9033: PageRuler Plus (Thermo Fisher Scientific); m385: Precision Plus Kaleidoscope (BioRad); Abcam (ab87438): Novex Sharp Prestained (Thermo Fisher Scientific). The immunoblots shown are representative of two separate experiments.

The article "Lack of specificity of antibodies raised against CLN3, the lysosomal/endosomal transmembrane protein mutated in juvenile Batten disease" was published in 2017. Journal: Biosci Rep.

We also tested several other anti-CLN3 antibodies in immunoblot experiments including the Q438 rabbit antibody raised against a peptide corresponding to amino acids 250–264 of human CLN3 [39], Q516 rabbit antibody raised against a human CLN3 peptide with amino acids 2–18 [37], rabbit antiserum 3326 against a GST-coupled human CLN3 peptide (amino acids 1–99) and its affinity-purified form, 33aff [35], rabbit antibodies 242 and 3787 raised against a keyhole limpet hemocyanin-coupled human CLN3 peptide (amino acids 242–258) and a GST-coupled human CLN3 peptide (amino acids 235–280) respectively [7,8], and five mouse monoclonal antibodies generated against two different CLN3 peptides by NeuroMab (UC Davis/NIH NeuroMab Facility). All these antibodies also lacked specificity, detected the same protein bands in WT samples as in *Cln3^−/−^* samples (data not shown).

## Discussion

Several studies examined the tissue expression and subcellular localization of CLN3, a putative lysosomal transmembrane protein, using various anti-CLN3 antibodies generated against either the whole CLN3 protein or short peptides from CLN3 [7,8,33–40]. The specificity of these antibodies, however, has never been verified with CLN3-deficient tissues or cells. In the present study, we tested the specificity of commercially available as well as researcher-generated anti-CLN3 antibodies using WT and *Cln3^−/−^* mouse tissue samples in immunoblot experiments. All the tested antibodies lacked specificity, they detected the same protein bands in wild-type and *Cln3^−/−^* samples.

The article "Lack of specificity of antibodies raised against CLN3, the lysosomal/endosomal transmembrane protein mutated in juvenile Batten disease" was published in 2017. Journal: Biosci Rep.

The 9033 rabbit anti-CLN3 serum we generated in our lab by immunizing with a peptide corresponding to amino acids 5–19 of mouse CLN3 was also not specific (Figure 5), neither was its immunogen affinity purified form (data not shown). This peptide was previously used by Ezaki et al. [50] to generate a rabbit anti-CLN3 antibody, and they showed by mass spectrometry that the protein band detected by this antibody contained CLN3. The mass spectrometry results, however, also indicated the presence of other proteins in the band [50]. Although we found that the Q438 rabbit antibody that was raised against a peptide corresponding to amino acids 250–264 of human CLN3 [39] did not detect a specific band in WT mouse tissue extracts as compared with *Cln3^−/−^* ones (data not shown), Chang et al*.* [51] showed the specificity of this antibody on an immunoblot with WT and *Cln3^−/−^* mouse whole brain extracts. However, they only presented a very narrow section of the blot without M.W. markers [51]. All the anti-CLN3 antibodies we tested were used either at the exact recommended concentration or within the recommended concentration range for immunoblotting (see Table 1). In the absence of detailed antibody dilution studies, however, we cannot rule out the possibility that some of the tested antibodies could display specificity for CLN3 at lower concentrations than recommended by the manufacturer.

A previous study has shown that a polyclonal antibody raised against a peptide antigen and anticipated to be specific to a low-voltage-activated calcium channel subunit also targeted neural cell adhesion molecule-180, and the cross-reactivity was due to a five-amino-acid epitope present in both proteins [52]. To examine if peptides used to generate anti-CLN3 antibodies contain motifs present in other proteins we performed Protein BLAST searches (NIH NCBI). The Abcam rabbit anti-CLN3 antibody (ab75959, Figures 1–4) was raised against a peptide corresponding to amino acids 400–438 (TSDEHREFAMAATCISDTLGISLSGLLALPLHDFLCQLS) of human CLN3. The Blast search using the first half (amino acids 400–419), second half (amino acids 420–438), or the middle (amino acids 416–424) of this sequence identified common short motifs in a number of different mouse (Mus musculus) proteins including a ubiquitin-associated and SH3 domain-containing protein A isoform (amino acids 170–178: REFAMA-AT), serine/threonine-protein kinase Sgk3 (amino acids 21–26: SDEHRE; amino acids 314–317: ISDT), mitochondrial antiviral-signaling protein isoform 2 (amino acids 99–109: A-AATC-S-TL), E74-like factor 3 (amino acids 1–8: MAATC-IS), mitogen-activated protein kinase kinase kinase 15 (amino acids 1069–1078: EHR MAAT IS), trace amine-associated receptor 5 (amino acids 84–90: GLL-LPL; amino acids 104–109: DFLC-L), fibrocystin precursor (amino acids 1784–1789: L-LPLH; amino acids 2524-2527: SLSG; amino acids 3171–3174: GLLA), leucine rich repeat containing protein 28 (amino acids 132–136: LLALP), nyctalopin precursor (amino acids 296–304: LSGLLAL-L), AP-5 complex subunit β-1 (amino acids 188–195: LLAL-LHD; amino acids 163–166: GLLA), stabilin 1 isoform (amino acids 83–87: ISLSG; amino acids 728–736: TLGIS-LSG), abnormal spindle-like microcephaly associated protein homolog (amino acids 3116–3121: DTLGIS), calmodulin-binding protein SHA1 (amino acids 569–574: DTLGIS), glycine decarboxylase isoform (amino acids 446–451: TLGISL), sodium/glucose cotransporter 2 (amino acids 539–544: TLGISL), and transmembrane protein 2 (amino acids 402–407: GISLSG).

The article "Lack of specificity of antibodies raised against CLN3, the lysosomal/endosomal transmembrane protein mutated in juvenile Batten disease" was published in 2017. Journal: Biosci Rep.

The 9033 rabbit anti-CLN3 serum (Figure 5) was generated in our lab by immunizing with a peptide corresponding to amino acids 5–19 (AGSWRRLEDSEREET) of mouse CLN3. This peptide was previously used by Ezaki et al. [50] to generate a rabbit anti-CLN3 antibody. The Blast search with amino acids 5–19 of mouse CLN3 found several mouse proteins containing sequence motifs of this peptide, such as α-actinin-2 (amino acids 394–397: RRLE), exosome component 9 isoform (amino acids 127–130: EREE; amino acids 266–273: LEDSE-EE), transmembrane protein 189 (amino acids 244–249: WRRLED), Map3k11 protein (amino acids 312–317: RRLEDS), mixed lineage kinase 3 (amino acids 551–556: RRLEDS), peroxisome proliferator activated receptor binding protein isoform (amino acids 13–16: GSWR; amino acids 32–36: EDSER), and golgin subfamily A member 4 (amino acids 518–526: RRLE–ERE; amino acids 1141–1144: SERE).

The Q438 rabbit anti-CLN3 antibody raised against a peptide corresponding to amino acids 250–264 of human CLN3 (RQPLIRTEAPESKPG) [39] has been used to examine the tissue expression and intracellular trafficking of endogenous CLN3 [37,38]. We tested this antibody in immunoblot experiments and it detected the same protein bands in WT samples as in *Cln3^−/−^* samples (data not shown). The Blast search with the peptide used to generate the Q438 anti-CLN3 antibody identified common short motifs in several human proteins including an ABI family member 3-binding protein isoform (amino acids 963–969: EAPESKP; amino acids 1029–1033: RTEAP), tubby-related protein 1 (amino acids 45–51: RTEAPES), plakophilin-4 isoform (amino acids 115–119: LIRTE), lysosome membrane protein 2 isoform 1 precursor (amino acids 132–135: LIRT; amino acids 472–478: R-PLIRT), lysosome membrane protein 2 isoform 2 precursor (amino acids 329–335: R-PLIRT), endoplasmin precursor (amino acids 690–695: R-PLIR), γ-adducin isoform a (amino acids 390–395: R-PLIR), transformation/transcription domain-associated protein isoforms (QPLIR); and also in several mouse (Mus musculus) proteins such as protein phosphatase Slingshot homolog 2 isoform 1 (amino acids 795–801: APESKPG) and isoform 2 (amino acids 801–807: APESKPG), trinucleotide repeat-containing gene 6A protein (amino acids 315–320: APESKP), retinoic acid receptor γ (amino acids 410–413: PLIR; amino acids 427–430: SKPG), and dipeptidase 2 isoform 1 precursor (amino acids 30–35: QPLI-T). The above findings provide a plausible explanation for the lack of specificity of anti-CLN3 antibodies.

The article "Lack of specificity of antibodies raised against CLN3, the lysosomal/endosomal transmembrane protein mutated in juvenile Batten disease" was published in 2017. Journal: Biosci Rep.

Because of the possible cross-reactivity to other proteins, the specificity of an antibody should always be checked using tissue samples from an appropriate knock-out animal or using knock-out cells. Our data provide evidence that immunization against a transmembrane protein with low to medium expression level does not necessarily generate specific antibodies.

## Abbreviations

BHK: baby hamster kidney
DDM: *n*-dodecyl-β-D-maltopyranoside
LCH: left cerebral hemisphere
M.P.: membrane proteins
M.W.: molecular weight
PVDF: polyvinylidene difluoride
RCH: right cerebral hemisphere
WT: wild type
